# Up-Regulation of pVHL along with Down-Regulation of HIF-1α by NDRG2 Expression Attenuates Proliferation and Invasion in Renal Cancer Cells

This article has been retracted.

**DOI:** 10.1371/journal.pone.0084127

**Published:** 2013-12-20

**Authors:** Lei Gao, Guo-jun Wu, Bei Liu, Ming-zhi Shen, Tie-jun Pan, Chui-gong Yu, Qin-hao Wang, Yi Ru, Xi-ping Liu, Tian-shui Niu, Guo-dong Wang, Ming Wei, Rui-xiao Li, Libo Yao, He Wang, Xia Li

**Affiliations:** 1 Department of Biochemistry and Molecular Biology, State Key Laboratory of Cancer Biology, the Fourth Military Medical University, Xi’an, China; 2 Department of Urology, Tangdu Hospital, the Fourth Military Medical University, Xi'an, China; 3 Department of Urology, Wuhan General Hospital, Guangzhou Command PLA, Wuhan, China; 4 Department of Urology, Xijing Hospital, the Fourth Military Medical University, Xi'an, China; 5 Department of Neurosurgery and Institute for Functional Brain Disorders, Tangdu Hospital, the Fourth Military Medical University, Xi'an, China; 6 Department of Cardiology, Hainan Branch of PLA General Hospital, Sanya, China; 7 Department of Urology, Armed Police General Hospital, Beijing, China; Eberhard-Karls University, Germany

## Abstract

The majority of renal cell carcinomas (RCCs) are characterized by loss of function of the tumor suppressor gene von Hippel Lindau (VHL), which acts as ubiquitin ligase for hypoxia-inducible factor-1α (HIF-1α). In the absence of VHL, HIF-1α protein becomes stabilized and contributes to tumorigenesis. Recent data demonstrate the antitumor efficacy of VHL promoter in RCC cells. This study demonstrates that N-Myc downstream-regulated gene 2 (NDRG2) is a potential regulator of VHL. NDRG2 is involved in proliferation and invasion of cancer cell, furthermore it is frequently down-regulated in renal cell carcinoma. Herein we evaluated the effect of NDRG2 overexpression on proliferation and invasion in human renal cancer cells. The human renal cancer cell line 786-O and A498 were infected with Ad-NDRG2 or Ad-LacZ. Overexpression of NDRG2 not only inhibited the growth of the cells, but also suppressed the invasion. Further study showed that the tumor suppressor gene VHL were up-regulated, whereas transcription factor HIF-1a and vascular endothelial growth factor (VEGF) were down-regulated in 786-O cells infected by Ad-NDRG2. Finally, in a nude mouse model, intratumoral injections of Ad-NDRG2 every 3 days for a total of seven times significantly inhibited the growth and angiogenesis of xenografted 786-O tumors. In conclusion, these data indicate that NDRG2 may be involved in proliferation and invasion by impacting the expression of VHL and HIF-1α. NDRG2 may be an attractive therapeutic target for renal cell carcinoma.

## Introduction

Renal cell carcinoma (RCC) is among the top 10 most common malignancies in both men and women [1]. RCC comprises a histologically diverse group of solid tumors, arising from different parts of the kidney [2]. The vast majority of RCCs are clear cell renal cell carcinomas (CCRCCs), characterized by loss of function of the tumor suppressor gene von Hippel Lindau (VHL). Defects in the VHL gene are the most common cause of familial CCRCC, and more than 80% of patients with sporadic CCRCC have an inactive VHL gene or loss of VHL gene[3]. 

VHL is a classical guardian inhibiting renal tumor initiation [4-6]. The protein VHL encoded by VHL gene, is a component of an E3 ubiquitin ligases complex that includes elongin-B, elongin-C, and cullin-2 [7,8]. Among the well-documented substrates of the pVHL is the hypoxia-inducible factor (HIF-1α), which is a transcription factor that controls the expression of hypoxia-induced factors such as pyruvate dehydrogenase kinase (PDK)-1, vascular endothelial growth factor (VEGF) and so on [9,10]. These target genes have influence on energy metabolism, cell proliferation and metastasis of CCRCC [11]. Under normal oxygen, HIF-1α binds pVHL through its hydroxylated proline residues and is polyubiquitinated by pVHL, which ultimately leads to the degradation of HIF-1α via the proteasome. During hypoxia, HIF-1α is not hydroxylated and escapes from pVHL-mediated degradation. The labile HIF-1α then forms functional transcription factor by associating with the constitutively expressed HIF-1β subunit [12]. Together, this complex binds to DNA motifs referred to as hypoxia response elements to regulate the expression of a number of genes involved in cell proliferation, metastasis and angiogenesis. Therefore, by promoting degradation of HIF-1α, pVHL can suppress HIF-1α stimulated transcription and function as a key tumor suppressor [13]. pVHL loss is a common event in CCRCC, leading to HIF-1α stabilization and the up-regulation of its target genes. It has been shown that VEGF expression is frequently elevated along with HIF-1α upregulation in many human cancers [14]. A previous study demonstrated that pVHL is able to enhance the expression and activity of another well-known tumor suppressor, p53 [14]. However, how pVHL itself is regulated has seldom been reported. Recent data have demonstrated the antitumor efficacy of a pVHL promoter in RCCs [15].

N-myc Downstream Regulated Gene 2 (NDRG2), is a member of the NDRG family, is a newly identified tumor suppressor. It has been reported that NDRG2 expression is downregulated in a variety of carcinomas, including liver cancer, pancreatic cancer, meningioma and prostate cancer. Studies from our lab and others have shown that NDRG2 is involved regulation of cell proliferation, apoptosis, differentiation and stress response [16-21]. Of note, our previous study implied that NDRG2 upregulated the expressions of p53 and pVHL while down-regulates the expressions of VEGF and HIF-1α in breast cancer cell lines [22]. Recently, it is reported that NDRG2 is downregulated in CCRCC tissues compared to adjacent non-neoplastic tissues [23]. Moreover, forced expression of NDRG2 inhibits the growth of clear cell RCC (CCRCC) cell lines and induces cell apoptosis [24]. These findings suggest that NDRG2 plays an important role in carcinogenesis of CCRCC. However, the exact role of NDRG2 in CCRCC is not fully understood. 

In this study, we attempted to explore whether there is a regulatory relationship between NDRG2 and pVHL. We first examined expression correlation between NDRG2 and pVHL in tumor tissues from CCRCC patients. Then we performed *in vitro* and *in vivo* experiments to investigate the effect of NDRG2 overexpression on cell behavior, as well as on the expression of pVHL and its downstream effectors, HIF-1α and VEGF. 

## Materials and Methods

### Ethics Statement

Human samples were obtained from all patients with written informed consent. Both written informed consent and study were approved by the Institutional Review Board of the Xijing Hospital, Fourth Military Medical University. The mice used in this research were obtained from the Fourth Military Medical University and were maintained at pathogen-free conditions. All procedures were done according to protocols approved by the Institutional Review Board of the Xijing Hospital, Fourth Military Medical University and conformed to the NIH guidelines on the ethical use of animals.

### Tissue collection and immunohistochemistry

A total of 130 formalin-fixed paraffin-embedded specimens of primary clear cell renal cell carcinoma and their adjacent normal kidney tissues were collected in the Department of Pathology of Xijing Hospital, Xi’an, China. All samples were obtained from patients who gave informed consent to use excess pathological specimens for research purposes. All patients provided written informed consent. The use of human tissues in this study was approved by the institutional review board of the Fourth Military Medical University and was conducted in accordance with international guidelines for the use of human tissues. Anti-NDRG2 (1:500 dilution) antibodies were purchased from BD Corporation (BD, NY, USA). Anti-HIF-1α (1:500 dilution) and anti-VEGF (1:1000 dilution) antibodies were from Santa Cruz Technology (Santa Cruz, CA, USA). Anti-VHL antibody (1:500 dilution) was from Neomarkers Corporation (Taipei, China). Anti-β-actin antibody (1:2000 dilution) was from Sigma (Sigma, USA). The immunohistochemistry kit was purchased from the Boster Company (Wuhan, CHN). 

The immunohistochemistry staining was performed according to the manufacturer’s instructions. Both the intensity and the extent of immunological staining were analyzed semi-quantitatively. Sections with no labeling or with fewer than 5% labeled cells were scored as 0. Sections were scored as a 1 if 5-25% of cells were labeled, as a 2 if 25-50% of cells were labeled, and as a 3 if 50-75% of cells were labeled. Finally, labeling of ≥75% of the cells was scored as a 4. The staining intensity was scored similarly, with 0 used for negative staining, 1 for weakly positive, 2 for moderately positive and 3 for strongly positive. The scores for the percentage of positive cells and for the staining intensity were multiplied to generate an immunoreactive score for each specimen. The product of the quantity and intensity scores were calculated such that a final score of 0 indicated no expression, 1-4 indicated weak expression, 5-8 indicated moderate expression and 9-12 indicated strong expression. The photos were collected through light microscopy (Olympus, Japan).

### Cell lines and reagents

Human renal cancer cell lines 786-O and A498 were obtained from the American Type Culture Collection (ATCC, USA). The cell lines were maintained in RPMI 1640 medium supplemented with 10% fetal bovine serum at 37 °C in a humidified incubator with 5% CO_2_. For hypoxia treatment, cells were cultured under hypoxic conditions (1% O_2_, 5% CO_2_ and 94% N_2_) and harvested at 24 h after infection.

### Cell growth assay

Cells were seeded (5 × 10^3^ cells per well) in triplicate in 96-well plates. After removing the medium, 40 MOI adenovirus expressing NDRG2 [24] or the negative control gene LacZ (Ad-LacZ) was added in serum-free RPMI 1640, incubated for 2 h, replaced with fresh RPMI 1640 supplemented with 10% FBS. Plates were then incubated for 0, 24, 48, and 72 h. The number of viable cells was determined using the 3-(4,5-dimethylthiazol-2-yl)-2,5-diphenyltetrazolium bromide (MTT) assay and reading the absorbance at 490 nm. The data are the mean ± standard deviation for three independent experiments. 

### Migration and invasion assays

Cell migration and invasion assays were done essentially as previously described [15]. Invasion assay with a Matrigel-coated membrane and migration assay with a Matrigel-uncoated membrane were performed using a 24-well chamber system (BD Biosciences, Bedford, MA), according to the manufacturer’s instructions. The cells were trypsinized and seeded in the upper chamber at 2.5×10^5^ cells/well in serum-free medium. The vector carrying LacZ or NDRG2, at a multiplicity of infection (MOI) of 40, was added immediately after cell plating. Medium supplemented with 5% FBS (used as a chemo-attractant) was placed in the bottom well. Incubation was carried out for 24 h at 37 °C in humidified air with a 5% CO_2_ atmosphere. The cells were allowed to migrate through a porous, Matrigel-coated or uncoated membrane (BD Biosciences). After the incubation, the chambers were removed, and invading cells on the bottom side of the membrane were fixed with methanol and stained with Gimsa. The number of invading cells or migrating cells were determined by counting five high-power fields (×400) on each membrane and calculated as the mean number of cells per field. The data are the mean ± standard deviation for three independent experiments.

### Western blotting analysis

Cells were seeded (5 × 10^5^ cells per well) in triplicate in 24-well plates. After removing the medium, 40 MOI Ad-NDRG2 or Ad-LacZ was added in serum-free RPMI 1640, incubated for 2 h, replaced with fresh RPMI 1640 supplemented with 10% FBS. After cultivating for 24 h, cells were washed with cold PBS and immediately lysed in a lysis buffer [1% Triton X-100,150 mmol/L NaCl, 100 mmol/L KCl, 20 mmol/L HEPES, 10 mmol/L EDTA, 1 mmol/L sodium orthovanadate, 10μg/ml aprotinin, 10 μg/ml leupeptin, and 1 μmol/L phenylmethylsulfonyl fluoride] on ice. Western blotting analysis was carried out according to the standard protocol using nitrocellulose membranes (Bio-Rad). For immunoblotting, membranes were incubated with the primary antibodies for overnight at 4°C, followed by 2 h incubation with a 1:2,000 dilution of horseradish peroxidase (HRP)-linked secondary antibody. Finally, the immunoreactive proteins were detected by the chemiluminescence detection system.

### Immunofluorescence assay

786-O cells were seeded on glass coverslips. After removing the medium, 40 MOI Ad-NDRG2 or Ad-LacZ was added in serum-free RPMI 1640, incubated for 2 h, replaced with fresh RPMI 1640 supplemented with 10% FBS. Plates were then incubated as described above for 24h. After permeabilization (0.5% Triton X-100), fixation (4% formaldehyde),and blocking (10% normal goat serum and 0.5% Triton X-100), mouse anti- NDRG2, VHL, HIF-1α and VEGF monoclonal antibody was added to cells for overnight at 4°C respectively. Cells were then stained with FITC-conjugated or Cy3-conjugated goat anti-mouse polyclonal antibody at 37 °C for 2 h in the dark. The fluorescence staining intensity was then examined by immunofluorescence microscopy. 

### ELISA

Cells were seeded (5 × 10^5^ cells per well) in triplicate in 24-well plates. After removing the medium, 40 MOI Ad-NDRG2 or Ad-LacZ was added in serum-free RPMI 1640, incubated for 2 h, replaced with fresh RPMI 1640 supplemented with 10% FBS. Conditioned media of the 24h cell cultures were assayed for VEGF by using commercial sandwich ELISA kits (Endogen, Woburn, MA, USA) according to manufacturer’s instructions. Each sample was tested in duplicate. Data were expressed in VEGF (pg /ml).

### Growth inhibition assays *in vivo*

 The Six-week-old BALB/C athymic (nu/nu) mice were provided by the Experimental Animal Center of the Fourth Military Medical University (Xi’an, China). All of the protocols were approved by the Animal Care and Use Committee at the Fourth Military Medical University and were performed in accordance with the animal care rules set forth by the university (Permit number: 10001). All efforts were made to reduce the number of animals used and to minimize their suffering. 786-O cells were harvested and resuspended in sterile PBS. 786-O cells (5 × 10^6^ cells) in 0.2 ml were injected subcutaneously into the left flanks of the 6-week-old nude mice. When the mean size of tumors reached 200 mm^3^, all the mice were divided into three groups randomly (Ad-NDRG2, Ad-LacZ and PBS Control groups, n = 10 per group). Intratumoral injections of adenovirus (1 × 10^9^ pfu in 100 ul PBS) were made every 3 d for a total of seven times. Tumor volumes were calculated based on caliper measurements of the length (a) and width (b) of the lesions using the following formula: V = ab^2^/2. The growth curve was then derived from these data. The conditions of the mice were monitored every day, and mouse survivals were recorded throughout the experimental period. The mouse was sacrificed by cervical dislocation, when it appeared cachexia, which was characterized as an overall state of ill health, accompanied by a loss of lean body mass and fat mass, weakness, fatigue, sluggishness, sharply decreased food intake, ascite and anorexia[25]. All sacrifices were performed under anesthesia (130 mg ketamine/8.8 mg xylazine/kg body weight). Then tumor specimens were removed to prepare paraffin sections for histological staining. The expression levels of NDRG2, pVHL, HIF-1α, VEGF protein in the inoculated tumors were detected using histology and immunohistochemistry as described above. 

### Statistical analysis

The statistical analyses were performed using SPSS software version 19.0. Comparisons between groups were undertaken using one-way ANOVA analysis and Fisher’s exact test. Kaplan-Meier curves and log-rank tests were used for the survival analysis. *P* < 0.05 was considered statistically significant.

## Results

### Expression of NDRG2, pVHL and HIF-1α in normal renal tissues and CCRCC tissues

To determine whether the regulation between NDRG2 and pVHL exists in CCRCC, we firstly detected the expression of NDRG2 and those of pVHL and HIF-1α in 130 CCRCC samples and the paired normal tissues. As is shown in Table 1 and Figure 1, the rate of NDRG2 positive expression in CCRCC tissue specimens was 30.0 % (Figure 1A and 1B), which was significantly lower than that in normal renal tissue 60.0 % (Figure 1G and 1H) (*P* =4.40 ×10^-9^). And the rate of pVHL positive expression in CCRCC tissue specimens (Figure 1C and 1D) was also significantly lower than that in normal renal tissue (Figure 1I and 1J) (26.9 % v.s. 66.2 %, *P* =3.02 ×10^-10^). On the contrary, the rate of HIF-1α positive expression in CCRCC tissue specimens (Figure 1E and 1F) was significantly higher than that in normal renal tissue (Figure 1K and 1L) (55.4 % v.s. 33.7 %, *P* =0.006). Furthermore, as is shown in Figure 1M and 1N , the expression levels of NDRG2 were positively correlated with those of pVHL in CCRCC tissue specimens (*r* = 0.749, *P* =3.25×10^-5^), while the expression levels of NDRG2 were negatively correlated with those of HIF-1α in CCRCC tissue specimens (*r* = -0.331, *P* =1.85×10^-3^).

**Table 1:** Expression of NDRG2, pVHL and HIF-1α in normal renal tissues and CCRCC tissues.

**Group**	**Subgroup**	**Negative(%)**	**Positive(%)**	^*χ*2^	***P* value**
NDRG2	CCRCC tissue	91(70.0)	39(30.0)	23.64	*P* =4.40 ×10^-9^
	normal renal tissue	52(40.0)	78(60.0)		
pVHL	CCRCC tissue	95(73.1)	35(26.9)	40.21	*P* =3.02 ×10^-10^
	normal renal tissue	44(33.8)	86(66.2)		
HIF-1α	CCRCC tissue	58(44.6)	72(55.4)	8.18	*P* =0.006
	normal renal tissue	81(62.3)	49(37.7)		

**Figure 1:** Expression of NDRG2, pVHL and HIF-1α in normal renal tissues and CCRCC tissues. Representative photomicrographs of immunohistochemical staining for NDRG2, pVHL and HIF-1αin normal renal tissues and CCRCC tissues. (A and B) NDRG2 expression in CCRCC tissues (200× magnification). (C and D) pVHL expression in CCRCC tissues (200× magnification). (E and F) HIF-1α expression in CCRCC tissues (200× magnification). (G and H) NDRG2 expression in normal kidney tubules (200× magnification). (I and J) pVHL expression in normal kidney tubules (200× magnification). (K and L) HIF-1αexpression in normal kidney tubules (200× magnification). (M) The expression levels of NDRG2 are positively correlated with those of pVHL. (N) The expression levels of NDRG2 are negatively correlated with those of HIF-1α. The number of specimen was shown as ‘scale’. Disparities across groups were analyzed using Pearson correlation coefficient and the graph was generated by SPSS19.0 software.

### NDRG2 overexpression inhibits proliferation of human renal cancer cells *in vitro*

To investigate the effects of NDRG2 overexpression on the growth of human renal cancer cells, we used Ad-LacZ or Ad-NDRG2 to infect 786-O cells and A498 cells. After infection for 24 h, strong expression of the NDRG2 protein in 786-O cells (Figure 2A) and A498 cells (Figure 2B) was confirmed by western blot analysis using a monoclonal antibody against NDRG2. Inhibition in cell proliferation was measured with the MTT assay 12, 24, 36, 48, 60 and 72 h following infection. As shown in Figure 2C and 2D, Ad-LacZ had no significant effect on cell proliferation in either cell lines compared with control group (*P* value at 24, 36, 48, 60 and 72 h is 0.55, 0.61, 0.96, 0.98 and 0.60 respectively in 786-O cells; *P* value is 0.60, 0.68, 0.60, 0.15 and 0.60 respectively in A498 cells). However, cell proliferation was significantly inhibited in Ad-NDRG2-infected 786-O cells (*P* value at 24, 36, 48, 60 and 72 h is 048, 1.54×10^-4^, 2.01×10^-4^, 2.15×10^-4^ and 4.32×10^-6^ respectively in 786-O cells) and Ad-NDRG2-infected A498 cells (*P* value is 0.47, 0.43, 2.20 ×10^-4^, 4.08 ×10^-4^ and 1.70 ×10^-6^ respectively in A498 cells), respectively, comparing to Ad-LacZ group.

**Figure 2:** Effect of NDRG2 on proliferation of renal cancer cells. (A and B) Expression levels of NDRG2 protein in Ad-NDRG2-infected 786-O and Ad-NDRG2-infected A498 cells were respectively examined by Western blotting. (C and D) The growth of the 786-O and A498 cells was inhibited by the overexpression of NDRG2 after 72 hours of incubation. Statistical significance was assessed using one-way ANOVA. *** indicates *P* < 0.001, when compared with the Ad-LacZ group.

### NDRG2 overexpression inhibits the invasion and migration of human renal cancer cells *in vitro*

To further evaluate the effect of NDRG2 overexpression on metastatic activity, we performed *in vitro* Matrigel-coated transwell invasion assays as well as migration assays with two different human renal cancer cell lines, 786-O and A498. Representative micrographs were taken from the lower surface of the transwell filter, and cells that invaded or migrated were stained with Gimsa. As shown in Figure 3A and 3B, the invasive potential, which is determined by the cells’ ability to invade a Matrigel barrier, was significantly suppressed by Ad-NDRG2 infection in 786-O cells (*P* =1.46×10^-5^ *v.s.* Ad- LacZ group) and A498 cells (*P* =2.23 ×10^-5^ *v.s.* Ad- LacZ group). However, there were no significant differences between Ad- LacZ group and control group in both 786-O cells (*P* =0.79) and A498 cells (*P* =0.58). Furthermore, overexpression of NDRG2 in these cell lines significantly suppressed their migration through the transwell when compared with Ad-LacZ infection (*P* =1.19 ×10^-5^ for 786-O cells and *P* =1.09 ×10^-3^ for A498 cells, respectively) (Figure 3C and 3D). But there were no significant differences between Ad- LacZ and control groups in both cell lines (*P* =0.73 for 786-O cells and *P* =0.94 for A498 cells)

**Figure 3:** Effect of NDRG2 on invasion and migration of renal cancer cells. (A and B) The invasion ability was estimated using Transwell coated with Matrigel. The amount of invaded cells was calculated in five random high-power fields (400×magnification). The histogram represents the quantification of cells that invaded. (C and D) The migration ability was estimated using Transwell uncoated with Matrigel. The amount of migrated cells was calculated in five random high-power fields (400× magnification). The histogram represents the quantification of cells that migrated. The data are the mean ± standard deviation (SD) for three independent experiments. Statistical significance was assessed using one-way ANOVA. ** or *** indicates *P* < 0.01 or *P* < 0.001, respectively, when compared with the Ad-LacZ group.

### Regulation of the expression of pVHL, HIF-1α and VEGF by up-regulation of NDRG2 in 786-O cells

 To understand the molecular mechanism through which NDRG2 inhibits 786-O cells proliferation and invasion, we analyzed the effect of NDRG2 on the expression of pVHL, HIF-1α and its target VEGF, which play important roles in cell proliferation and invasion in renal cancer. We infected the 786-O cells with Ad-NDGR2 and examined pVHL, HIF-1α and VEGF expression by western blot analysis. As a result, we disclosed the increased pVHL expression and reduced HIF-1α and VEGF in comparison to that of control group and Ad-LacZ group 786-O cells (Figure 4A). Meanwhile, we used immunofluorescence assay to further affirm regulation of the expression of pVHL, HIF-1α and VEGF by overexpression of NDRG2. Indirect immunofluorescence labeling showed weak signals of NDRG2 and pVHL in control group and Ad-LacZ group 786-O cells, whereas there was stronger staining of NDRG2 and pVHL in Ad-NDRG2-infected 786-O cells. Moreover, the signals of HIF-1α and VEGF in control and Ad-LacZ group were stronger than those in Ad-NDRG2 group (Figure 4B). 

**Figure 4:** Effect of NDRG2 on the expression of pVHL, HIF-1α and VEGF under normoxia or hypoxia. (A) 786-O, Ad-LacZ-786-O and Ad-NDRG2-786-O cells were incubated under normoxia and hypoxia for 24 h. After incubation, the cells were analyzed by western blot assay. β-actin protein levels were used as a loading control. (B) After infection of 786-O cells with 40 MOI Ad-NDRG2 under normoxia for 24 h, protein levels of NDRG2, pVHL, HIF-1α and VEGF in the cells were measured using immunofluorescence assay (400× magnification).

### VEGF production is inhibited by NDRG2 overexpression

To test whether NDRG2 expression affects the VEGF production in renal cancer cells, we used Ad-NDRG2 to infect 786-O and A498 cells and measured the VEGF levels in cell culture medium under normoxic or hypoxic conditions. The results of ELISA assay showed that Ad-NDRG2 group of 786-O cells, as compared to Ad-LacZ exhibited significantly decreased VEGF secretion under either normoxic (Figure 5A) (*P* =7.32 ×10^-8^) or hypoxic conditions (Figure 5B) (*P* =9.95 ×10^-8^). Meanwhile, the VEGF secretion of A498 cells was also significantly decreased under NDRG2 overexpression condition irrespective of normoxia (Figure 5C) (*P* =6.12 ×10^-7^) and hypoxia (Figure 5D) (*P* =0.005). But Ad-LacZ infection has no effect on VEGF production compared with control group either in normoxia (*P* =0.55 for 786 O cells; *P* =0.91 for A498 cells) or in hypoxia (*P* =0.94 for 786 O cells; *P* =0.90 for A498 cells).

**Figure 5:** Effect of Ad-NDRG2 on VEGF secretion in renal cancer cells under normoxia or hypoxia. (A and B) 786-O, Ad-LacZ-786-O and Ad-NDRG2-786-O cells were incubated under normoxia and hypoxia for 24 h. After incubation, the media were analyzed for VEGF levels by ELISA assay. (C and D) A498, Ad-LacZ- A498 and Ad-NDRG2- A498 cells were incubated under normoxia and hypoxia for 24 h. After incubation, the media were analyzed for VEGF levels by ELISA assay. The data were the mean ± standard deviation (SD) for three independent experiments. Statistical significance was assessed with one-way ANOVA. ** or *** indicates *P* < 0.01 or *P* < 0.001, respectively, when compared with the Ad-LacZ group.

### Suppression of tumor growth in a nude mouse model by intratumoral injection of Ad-NDRG2

To investigate the effects of Ad-NDRG2 on tumor growth *in vivo*, we injected adenovirus (1 x 10^9^ pfu in 100 ul PBS) Ad-NDRG2, Ad-LacZ or PBS every 3 days into pre-established human 786-O renal cancer tumors (approximately 200 mm^3^) grown in nude mice. As shown in Figure 6A, the Ad-NDRG2 group achieved a sustained and significant inhibition of tumor growth compared with Ad-LacZ group (*P* value is 0.002, 1.54 ×10^-6^, 1.77 ×10^-6^, 9.7 ×10^-11^, 8.69 ×10^-12^ and 1.35 ×10^-9^ at Day6, 9, 12, 15, 18 and Day 21 respectively). Kaplan-Merier survival analysis showed that intratumoral injection of Ad-NDRG2 significantly prolonged mice survival times (*χ* ^2^ =11.75, *P* = 0.003) (Figure 6B). No significant differences were observed between control group and Ad-LacZ group (*χ* ^2^=4.67, *P*=0.122), and the results were consistent with those of the *in vitro* assays. After the mice were sacrificed, the tumors were removed for analysis of the expression of NDRG2, pVHL, HIF-1α and VEGF. Immunolabeling for VEGF and HIF-1a were lower in tumors excised from mice in the Ad-NDRG2 group. Moreover, the NDRG2 and pVHL expression levels in the Ad-NDRG2 group were dramatically increased while HIF-1α and VEGF levels decreased compared to Ad-LacZ group (NDRG2, *P* =6.47 ×10^-8^; pVHL, *P* =1.55 ×10^-8^; HIF-1α, *P* =0.0001; VEGF, *P* =6.07 ×10^-7^). There was no significant difference between the control and Ad-LacZ groups (NDRG2, *P* =0.98; pVHL, *P* =0.94; HIF-1α, *P* =0.78; VEGF, *P* =0.69) (Figure 7A and 7B). 

**Figure 6:** Effects of Ad-NDRG2 intratumoral injections on tumor growth and long-term survival of 786-O cells tumor-bearing mice. (A) Tumor growth curve. The tumor growth was assessed every 3 days until Day 21 of treatment by measuring two perpendicular diameters and calculating the volume in mm^3^. Statistical analysis was assessed with one-way ANOVA. ** or *** indicates P < 0.01 or P < 0.001 when compared with the Ad-LacZ group. (B) Kaplan–Meier curve was shown in the Control, Ad-LacZ and Ad-NDRG2 groups, with each group consisting of ten mice. There was a significant difference between Ad-NDRG2 and Ad-LacZ treatments. Statistical significance was assessed using log-rank tests. ** indicates *P* < 0.01 when compared with the Ad-LacZ group.

**Figure 7:** Effects of Ad-NDRG2 intratumoral injections on NDRG2, pVHL, HIF-1α and VEGF expression of 786-O cell xenografts in mice. (A) Intratumoral expressions of NDRG2, pVHL, HIF-1a and VEGF were assessed by Immunohistochemistry (200× magnification) on paraffin-embedded 786-O cell tumor sections. Representative images are shown. (B) Integrated optical density (IOD) values of NDRG2, pVHL, HIF-1α and VEGF protein expression of the tumors were evaluated. ImagePro Plus software was utilized to analyze the IOD values of the positive areas of immunohistochemical staining, and the resulting histograms are shown. Statistical analysis was carried out using one-way ANOVA. The results were shown as the mean ± SD. ***P < 0.001.

## Discussion

Though surgical resection and adjuvant therapy are commonly used to treat renal cancer patients, the overall survival rate for renal cancer requires improvement. It is known that RCC is resistant to radio-, hormono-, and chemotherapy [26]. Therefore, the development of biological therapies for renal cancer is urgently needed. The occurrence and development of renal cancer depends upon the expression of several related genes, such as HIF-1α, PDK1, VEGF and so on [27]. 

Multiple studies have now demonstrated that HIF-1α up-regulates the expression of PDK1 and VEGF[28]. Moreover, PDK1 and VEGF expression are increased in RCC [29,30]. PDK1 is known to phosphorylate and activate some protein kinases that belong to the AGC family of protein kinases. One of the protein kinases is protein kinase B (PKB, also known as Akt). PDK1 activates Akt by phosphorylating a Ser/Thr residue in the activation loop. Akt pathway is aberrantly activated in CCRCC and involved in the proliferation and metastasis [31]. And VEGF is the mainstay amid all angiogenic factors and promotes both tumorigenesis and invasion of RCC [32]. HIF-1α are also frequently overexpressed in renal cancer, which correlate with poor clinical prognosis [33]. Since elevated HIF-1α expression up-regulates the expression of PDK1 and VEGF, which promotes tumor progression. So the inhibition of HIF-1α expression is a promising approach to treat renal cancer. This strategy might be especially effective against RCCs that have constitutive HIF-1α activity due to the loss of pVHL expression. 

The present data have implied that NDRG2 expression was downregulated or lost in several malignant tumors compared to normal or benign tissues, suggesting that NDRG2 plays a crucial role in carcinogenesis and tumor progression [34]. In our prophase study, it was shown that NDRG2 expression is decreased in human CCRCC tissues and cell lines compared with matching adjacent non-tumoral tissue and normal renal cell lines [23]. It was also shown that NDRG2 down-regulation is associated with advanced and aggressive tumor behaviors that are relevant to tumor metastasis and survival in CCRCC [35]. So the identification of NDRG2 as an important regulator of tumor cell migration and invasion *in vitro* emphasizes an essential role of this NDRG2 in mediating renal oncogenesis and tumor behavior. What is more, NDRG2 may be a novel target for future biological therapies for renal cancer. Recently, some reports demonstrate that infection by Ad-NDRG2 reduced HIF-1α and VEGF expression in breast cancer cells [22]. 

In this paper, our data revealed that NDRG2 overexpression in renal cancer cells could suppress 786-O and A498 cells proliferation and invasion. Importantly, tumor growth in a nude mouse model was inhibited by intratumoral injection of Ad-NDRG2. This effect may be related to the up-regulation of pVHL and down-regulation of HIF-1α. Both *in vitro* and *in vivo* overexpression of NDRG2 by Ad-NDRG2 in 786-O cells can increased pVHL expression and decreased HIF-1α and VEGF expression. And it is possible that the NDRG2-overexpression-caused down-regulation of HIF-1α and VEGF is partly due to up-regulation of the tumor suppressor genes VHL. Forced expression of NDRG2 may regulate pVHL either in transcriptional level or in protein degradation level, which will be further clarified in our future study. We also cannot exclude the possibility that NDRG2 regulate HIF-1α expression and consequent VEGF changes independent of pVHL, because a previous study reported that ectopic NDRG2 expression leads to p53 elevation, which is another HIF-1α regulator. Moreover, the more complicated interplay between NDRG2, pVHL and HIF-1α may co-exist in CCRCC. It is reported that the loss of pVHL is associated with modulations of the TGF-β1, whose expression is correlated to poor prognosis in CCRCC [36-39], while NDRG2 can antagonize TGF-β1 mediated tumor cell invasion in hepatocellular carcinomas [40]. Another report showed that pVHL is a negative regulator of Nuclear Factor kappa B (NF-kappa B). The loss of pVHL has been associated with enhanced NF-kappa B expression and activity in CCRCC [41]. Meanwhile, some reports showed that NDRG2 affects malignant mouse melanoma cell invasion by suppressing NF-kappa B activity [42]. Therefore, the two tumor suppressor, pVHL and NDRG2 may converge into the same signaling pathways or downstream effectors and control CCRCC malignancy. Together, ectopic expression of NDRG2 is a powerful anti-tumor strategy, antagonizing HIF-1α-VEGF axis either directly or indirectly by regulating pVHL (Figure 8).

**Figure 8:** Proposed model that NDRG2 exerts its anti-tumor effect. The NDRG2 caused down-regulation of HIF-1α and VEGF was partly due to up-regulation of the tumor suppressor pVHL. It could not be excluded that NDRG2 may also regulate HIF-1α expression and consequent VEGF changes independent of pVHL.

In summary, NDRG2 could inhibit human renal cancer cell proliferation and invasion by itself or by affecting HIF-1α mediated processes. Further exploration on the molecular mechanism of NDRG2 modulation may offer a novel approach for treating human renal cancer. Especially, targeting NDRG2 may be an effective means of treating human renal cancer of pVHL expression loss.
